RETRACTED

# Effect of Combined Spinal-Epidural Anesthesia and Total Intravenous Anesthesia on Hemodynamics and Pregnancy Outcomes of Severe Preeclampsia Pregnant Patients Undergoing Cesarean Section

**DOI:** 10.1155/2022/2655858

**Published:** 2022-02-22

**Authors:** Guangrong Wang, Pengyu Zhang, Minghui Li, Xiujuan Wu, Hua Li

**Affiliations:** ^1^Department of Operating Room of Anesthesiology, Zaozhuang Traditional Chinese Medicine Hospital, Beijing University of Chinese Medicine Zaozhuang Hospital, Beijing University of Chinese Medicine Fourth Clinical Medicine College, Zaozhuang 277000, Shandong, China; ^2^The Second Department of Internal Medicine-Neurology, Zhangqiu District People's Hospital, No. 1920 Mingshui Huiquan Road, Zhangqiu, Jinan 250200, Shandong, China; ^3^Department of Obstetrics, Taian Maternal and Child Health Hospital, Taian 271000, Shandong, China; ^4^Department of Outpatient, Taian Maternal and Child Health Hospital, Taian 271000, Shandong, China; ^5^Department of Obstetrics, Zhangqiu District People's Hospital, Jinan 250200, Shandong, China

## Abstract

**Objective:**

The purpose of the study was to investigate the effect of combined spinal-epidural anesthesia (CSEA) and total intravenous anesthesia (TIVA) on hemodynamics and pregnancy outcomes of severe preeclampsia pregnant patients undergoing cesarean section.

**Methods:**

126 patients with severe preeclampsia admitted to Zhangqiu District People's Hospital from August 2018 to August 2019 were selected as the study subjects and randomly divided into the experimental group (*n* = 63) and control group (*n* = 63). After undergoing cesarean section, the patients in the experimental group received CSEA, while those in the control group were given TIVA. After that, the effect of different anesthesia methods on the hemodynamics and pregnancy outcomes of pregnant women was compared.

**Results:**

There were no significant differences in age, BMI value, weight, height, gestational weeks, SBP, DBP, and residence between the two groups (*P* > 0.05). The operation duration, the onset time of anesthesia, and delivery time in the experimental group were significantly shorter than those in the control group, with less intraoperative blood loss in the experimental group than that in the control group (*P* < 0.001). In both groups, MAP and SpO_2_ during delivery were significantly lower than those before anesthesia, and HR was significantly higher than that before anesthesia (*P* < 0.001). In the experimental group, MAP and HR during delivery were significantly lower than those in the control group, and SpO_2_ was significantly higher than that in the control group (*P* < 0.001). The total effective rate of anesthesia in the experimental group was significantly higher than that in the control group (*P* < 0.05). The Apgar scoring of the newborns in the experimental group was significantly higher than that in the control group (*P* < 0.001), and the total incidence of postoperative adverse reactions in the experimental group was significantly lower than that in the control group (*P* < 0.05).

RETRACTED

**Conclusion:**

CSEA is a reliable anesthesia method for improving the hemodynamics indicators in pregnant patients with severe preeclampsia; such strategy greatly increases the Apgar score of newborns and shortens the anesthesia onset time. Further research will be conducive to establishing a better anesthesia plan for such patients.

## 1. Introduction

Preeclampsia, a common pregnancy complication mostly occurring after 20 weeks of gestation, is mainly manifested by elevated blood pressure and proteinuria. With the progress of the disease, severe preeclampsia will further develop into eclampsia, which results in convulsions or coma of puerperae and induces some complications such as heart failure, retinal detachment, and placental abruption, seriously threatening maternal and infant health [1, 2]. The latest data from the World Health Organization showed that the incidence of severe preeclampsia was 3.2–5% and the death rate was 4.3–5.6% [3]. At present, cesarean section is a common treatment for severe preeclampsia, and the selection of anesthesia methods has become the research focus of current medical community. CSEA has the advantages of the rapid onset time, good blocking effect, and obvious analgesic effect, which have been proven in patients with pregnancy-induced hypertension syndrome undergoing cesarean section [4]. TIVA refers to the adoption of multiple short-acting intravenous anesthetics after the induction of routine intravenous anesthesia to maintain anesthesia in the form of intermittent or continuous intravenous injection, with the effect that has been confirmed in elderly patients undergoing abdominal operation [5]. However, prolonged TIVA easily causes drug accumulation in the body and extends awakening time and has the possibility of triggering circulatory depression, leading to conduction disturbances in the heart and susceptibility to arrhythmias. Different anesthesia methods bring different effects to pregnant women and pregnancy outcomes [6]. Whether the abnormal changes of hemodynamics in blood pressure during anesthesia aggravates pregnant patients' conditions and adversely affects surgery becomes an important issue for anesthesiologists to take into account [7]. Currently, there are few reports exploring the application of CSEA and TIVA in severe preeclampsia pregnant patients undergoing cesarean section. Based on that, in this study, with the purpose of further exploring the effect of CSEA and TIVA on hemodynamics and pregnancy outcomes of severe preeclampsia pregnant patients undergoing cesarean section, 126 pregnant patients with severe preeclampsia admitted to Zhangqiu District People's Hospital from August 2018 to August 2019 were selected as the study subjects, and the summary report is as follows.

RETRACTED

## 2. Materials and Methods

### 2.1. General Information

126 patients with severe preeclampsia admitted to Zhangqiu District People's Hospital from August 2018 to August 2019 were selected as the study subjects and randomly divided into the experimental group (*n* = 63) and control group (*n* = 63). The study met the World Medical Association Declaration of Helsinki [8].

### 2.2. Inclusion Criteria

The inclusion criteria were as follows: patients met the diagnostic criteria for severe preeclampsia, i.e., systolic blood pressure ≥160 mmHg, diastolic blood pressure ≥110 mmHg, platelet count <1 × 10^6^, or the occurrence of kidney function impairment, pulmonary edema, and visual disorder, and their clinical manifestations included dizziness, vomiting, abdominal distention, and palpitation; patients met the indications of cesarean section and had single birth; and patients had no other pregnancy complications. This study was approved by the Ethics Committee of Zhangqiu District People's Hospital, and pregnant patients and their families were informed of the purpose and process of this study and signed the informed consent.

### 2.3. Exclusion Criteria

The exclusion criteria were as follows: patients had organic lesions in the brain, heart, lungs, and kidneys; patients had abnormal systemic coagulation; patients had contraindications to surgery or anesthesia; and patients had cognitive impairment such as mental disorders or refused to cooperate with the study.

### 2.4. Methods

In the control group, the patients received TIVA with the intravenous injection of 1.5 mg/kg of propofol (State Food and Drug Administration approval number: H20093542; manufacturer: Hebei Yipin Pharmaceutical Co., Ltd.; specification: 10 ml: 0.1 g). When the onset of anesthesia was observed, the patients were injected intravenously with 0.6 mg/kg of rocuronium bromide (State Food and Drug Administration approval number: H20100069; manufacturer: Hebei Baiqi Pharmaceutical Co., Ltd.; specification: 5 ml: 50 mg) and 1.0 *μ*g/kg of remifentanil (State Food and Drug Administration approval number: H20030197; manufacturer: Yichang Humanwell Pharmaceutical Co., Ltd.; specification: 1 mg). Before delivery, the patients underwent pump infusion of propofol at 2.5 mg/kg per hour and remifentanil at 0.05 mg/kg per minute at the same time. After the birth of the newborns, the continuous pump infusion of 0.05 mg/kg of midazolam (State Food and Drug Administration approval number: H10980026; manufacturer: Jiangsu Nhwa Pharmaceutical Co., Ltd.; specifications: 3 ml: 15 mg) and 0.3 mg/kg of sufentanil (State Food and Drug Administration approval number: H20054172; manufacturer: Yichang Humanwell Pharmaceutical Co., Ltd.; specification: 2 ml: 100 *μ*g) were performed at 3-4 mg/kg per hour, and 0.2 mg/kg of rocuronium was also added to maintain anesthesia [9].

RETRACTED

In the experimental group, the patients were treated with CSEA. Epidural puncturing was carried out in pregnant patients' intervertebral space from L_2_ to L_4_, and lumbar puncture was performed with puncture needles by routine techniques of needling. After cerebrospinal fluid flowed out, the patients were injected with 1.2 ml of 0.75% levobupivacaine (State Food and Drug Administration approval number: H20050403; manufacturer: Zhuhai Rundu Pharmaceutical Co., Ltd.; specification: 5 ml: 37.5 mg) for 10 s. After withdrawing the needles, tubes were inserted in epidural space, and then, the patients took supine positions. Subsequently, the intravenous injection with 5 ml of 2% lidocaine hydrochloride injection (State Food and Drug Administration approval number: H44023825; manufacturer: Guangzhou Baiyunshan Mingxing Pharmaceutical Co., Ltd.; specification: 2 ml: 40 mg) was conducted to the patients; if the signs of subarachnoid space anesthesia were not observed after 5 minutes of injection, the patients were injected with 5 ml of bupivacaine hydrochloride injection (State Food and Drug Administration approval number: H37022107; manufacturer: Shandong Hualu Pharmaceutical Co., Ltd.; specification: 5 ml: 37.5 mg) and 5 ml of 2% lidocaine. When the anesthesia was maintained at level T8, the cesarean section was carried out.

### 2.5. Evaluation Indexes

The operation duration, the onset time of anesthesia, delivery time, and intraoperative blood loss were recorded in both groups.

Mean arterial pressure (MAP), heart rate (HR), and oxygen saturation (SpO_2_) before anesthesia and at delivery were measured in both groups. MAP = (systolic blood pressure + 2 × diastolic blood pressure)/3; the HR value was measured by the electronic sphygmomanometer (manufactured: Nanjing Vedeng Medical Co., Ltd.); and SpO_2_ was measured by the fingertip photoelectric sensor (manufactured: Guangzhou Sichuang Hongyi Electronic Technology Co., Ltd.), during which the pregnant patients were told to keep the body relaxed while the sensor was clamping to their fingertips.

RETRACTED

The condition that after anesthesia, with appropriate muscle relaxation, the patients had no adverse reactions during the surgery which was carried out smoothly was excellent; the condition that after anesthesia, with good muscle relaxation, the patients had slight tremors during the surgery, which did not affect the surgery was effective; the condition that after anesthesia, with poor muscle relaxation, the patients had significant tremors after the surgery, and they should be given analgesic and sedative drugs to finish the surgery and was ineffective. The total effective rate = (number of excellent cases + number of effective cases)/total number of cases × 100%.

The newborns' physical conditions in both groups were evaluated by referring to the Apgar scoring [10], with the total score of 10 points. 7–10 points represented normal condition, 4–7 points represented mild asphyxia, and 4 points and below represented severe asphyxia. The scoring items included color of the skin, breathing, reflection, heartbeat rate, muscle tone, and movement.

Postoperative adverse reactions were recorded in both groups, including hypotension, pulmonary edema, and traction reaction.

### 2.6. Statistical Methods

The data in the study were statistically analyzed and processed by SPSS 21.0 software. GraphPad Prism 7 (GraphPad Software, San Diego, USA) was used to draw pictures of the data. Measurement data were expressed by (±*s*) and tested by the *t*-test. Enumeration data were expressed as (*n* (%)) and tested by the *X*^2^ test. The differences had a statistical significance when *P* < 0.05.

## 3. Results

### 3.1. Comparison of Clinical Data between the Two Groups

There were no significant differences in age, BMI value, weight, height, gestational weeks, SBP, DBP, and residence between the two groups (*P* > 0.05), which were comparable, as given in Table 1.

### 3.2. Comparison of Surgical Conditions between the Two Groups

The operation duration, the onset time of anesthesia, and delivery time in the experimental group were significantly shorter than those in the control group, and the intraoperative blood loss in the experimental group was significantly less than that in the control group (*P* < 0.05), as given in Table 2.

### 3.3. Comparison of Hemodynamic Indexes at Different Time Points between the Two Groups

In both groups, MAP and SpO_2_ at delivery were significantly lower than those before anesthesia, and HR at delivery was significantly higher than that before anesthesia (*P* < 0.05). MAP and HR at delivery in the experimental group were significantly lower than those in the control group, and SpO_2_ in the experimental group was significantly higher than that in the control group (*P* < 0.05), as given in Table 3.

RETRACTED

### 3.4. Comparison of the Anesthetic Effect between the Two Groups

The total effective rate of anesthesia in the experimental group was significantly higher than that in the control group (*P* < 0.05), as given in Table 4.

### 3.5. Comparison of Apgar Scoring between the Two Groups

The Apgar scoring of newborns in the experimental group was significantly higher than that in the control group (*P* < 0.05), as shown in Figure 1.

The Apgar scoring of the newborns in the experimental group was (9.28 ± 0.33) points, while that in the control group was (8.41 ± 0.86) points.

^*∗*^Significant difference in Apgar scoring between the two groups (*t* = 7.497, *P* < 0.001).

### 3.6. Comparison of Adverse Reactions after Surgery between the Two Groups

The total incidence of postoperative adverse reactions in the experimental group was significantly lower than that in the control group (*P* < 0.05), as given in Table 5.

## 4. Discussion

Preeclampsia is one of the peculiar diseases of pregnancy, characterized by disorders of uterine spiral artery remodeling, endothelial damage, and local ischemia as the basic pathological changes [11]. Parturient presents with preeclampsia present systemic inflammatory response, mainly manifesting clinically as edema, hypertension, and proteinuria. Severe eclampsia is severe and sudden in onset, and affected women generally experience headaches with syncope and unconsciousness, which can lead to generalized arteriolar spasms, local ischemia, endothelial damage, and resultant blood supply deficiency of tissue and organs, and in severe cases, maternal and fetal death [12]. Research investigations have shown [13] that the number of maternal deaths from eclampsia greatly exceeds 100,000 per year in China. As severe preeclampsia can easily progress to eclampsia and its condition is difficult to control, the pregnant patients have to receive cesarean section immediately to terminate pregnancy; thus, the selection of anesthesia methods is essential for the implementation of surgery [14, 15]. Generally speaking, the hospitals mostly carry out CSEA for cesarean section because it can quickly make the pregnant patients enter anesthesia states, with longer time of blocking and a better therapeutic effect [16, 17]. TIVA is a type of anesthesia that completely relies on intravenous injection or infusion of anesthetics to finish surgery, which easily leads to respiratory depression and circulation inhibition, greatly increasing the surgical risks. Besides, propofol, rocuronium, and other drugs used in anesthesia will increase the patients' pains, adversely affecting surgery [18, 19].

RETRACTED

Clinical studies have confirmed that CSEA can make the human body enter optimal anesthesia states without large doses of anesthetics. During the process of anesthesia, drug doses can be adjusted appropriately according to maternal delivery conditions [20]. Severe preeclampsia is mostly caused by the imbalance of the maternal immune system, placental calcium deficiency, or ischemia; hence, the implementation of effective anesthesia can further improve maternal physical health and increase the neonatal survival rate. This study confirmed that the total effective rate of CSEA in the experimental group was significantly higher than that in the control group (*P* < 0.05), which was presumably related to the lower dosage of this anesthesia, leading to the surgical requirements for muscle relaxation and the less impact on its hemodynamics. This study found that the incidence of adverse reactions in the experimental group was significantly lower than that in the control group (*P* < 0.05). Clendenon et al. [21] pointed out that the incidence of adverse reactions in patients undergoing cesarean section was 4.53%, which was significantly lower than 16.03% in the reference group (*P* < 0.05), demonstrating that the purpose of this study was to show that CSEA could significantly reduce the adverse reactions after cesarean section and improve maternal and infant health. It was speculated that the results might be correlated with the administration methods of CSEA, where the administration was performed in external cavity and lumbar puncture was conducted with fine puncture needles, effectively reducing the clinical adverse reactions of pregnant patients after surgery. Academic studies have also revealed that CSEA can maintain the stability of maternal hemodynamics, reduce heart rate fluctuation, improve blood supply, and reduce surgical risks [22, 23]. The limitations of the study: based on the limited study area, the sample size selected was only the patients within our region and did not include those from other regions, so the results obtained may be affected by factors such as the small sample size and region.

In conclusion, CSEA can make the hemodynamics of severe preeclampsia pregnant patients undergoing cesarean section in stable states, improve the delivery outcomes, and reduce the adverse reactions after surgery, with a better anesthetic effect, which is worthy of application and popularization.

## Figures and Tables

**Figure 1:** Comparison of Apgar scoring between the two groups (±*s*). The abscissa represents the experimental group and control group, while the ordinate represents Apgar scoring.

RETRACTED

**Table 1:** Comparison of clinical data between the two groups.

Types	Experimental group (*n* = 63)	Control group (*n* = 63)	*χ* ^2^ (*t*)	*P*
Average age (years old)	28.17 ± 0.63	28.14 ± 0.65	0.263	0.793
BMI (kg/m^2^)	21.53 ± 1.25	21.55 ± 1.26	0.089	0.929
Weight (kg)	69.21 ± 2.43	69.24 ± 2.45	0.069	0.945
Height (cm)	162.45 ± 3.65	162.52 ± 3.67	0.107	0.915
Gestational weeks (weeks)	34.85 ± 1.25	34.86 ± 1.28	0.044	0.965
SBP (mmHg)	174.25 ± 2.43	174.27 ± 2.42	0.046	0.963
DBP (mmHg)	125.24 ± 2.21	125.26 ± 2.24	0.050	0.960
Residence			0.032	0.858
Urban area	28 (44.44%)	29 (46.03%)		
Rural area	35 (55.56%)	34 (53.97%)		

**Table 2:** Comparison of surgical conditions between the two groups (±*s*).

Group	*n*	Operation duration (min)	The onset time of anesthesia (min)	Delivery time (min)	Intraoperative blood loss (ml)
Experimental group	63	42.14 ± 7.64	6.25 ± 1.85	12.32 ± 5.78	142.54 ± 18.77
Control group	63	51.55 ± 7.58	11.58 ± 1.69	25.44 ± 5.49	185.31 ± 18.64
*t*		6.940	16.884	13.063	12.833
*P*		0.001	0.001	0.001	0.001

**Table 3:** Comparison of hemodynamic indexes at different time points between the two groups (±*s*).

Group	*n*	Time	MAP (mmHg)	HR (time/min)	SpO_2_ (%)
Experimental group	63	Before anesthesia	123.25 ± 4.26	78.77 ± 1.65	95.21 ± 2.08
		At delivery	97.43 ± 3.18	80.32 ± 1.73	93.18 ± 1.28

Control group	63	Before anesthesia	123.28 ± 4.29	78.79 ± 1.69	95.24 ± 2.06
		At delivery	105.22 ± 3.15^∗^	87.22 ± 1.83^*∗*^	90.63 ± 1.32^*∗*^

Each hemodynamic index at delivery in both groups was significantly lower than that before anesthesia; ^*∗*^comparison between the experimental group and the control group, *P* < 0.001.

**Table 4:** Comparison of the anesthetic effect between the two groups (*n* (%)).

Group	*n*	Excellent	Effective	Ineffective	Total effective rate
Experimental group	63	24 (38.10%)	37 (58.73%)	2 (3.17%)	96.83% (61/63)
Control group	63	19 (30.16%)	35 (55.56%)	9 (14.29%)	85.71% (54/63)
*X* ^2^					4.881
*P*					<0.05

**Table 5:** Comparison of adverse reactions between the two groups (*n* (%)).

Group	*n*	Hypotension	Pulmonary edema	Traction reaction	Total incidence
Experimental group	63	1 (1.59%)	0 (0.00%)	2 (3.17%)	4.76% (3/63)
Control group	63	3 (4.76%)	3 (4.76%)	4 (6.35%)	15.87% (10/63)
*X* ^2^					4.203
*P*					0.040

## Data Availability

The data used to support the findings of this study are available from the corresponding author upon request.
